RETRACTED

# Contemporary Value Assessment of Marxist Ideology under the Context of Deep Learning

**DOI:** 10.1155/2022/4654153

**Published:** 2022-06-15

**Authors:** Jian Sun

**Affiliations:** ^1^School of Marxism, Nanjing University of Aeronautics and Astronautics, Nanjing Jiangsu 211170, China; ^2^School of Marxism, Jiangsu Maritime Institute, Nanjing Jiangsu 211170, China

## Abstract

As a conceptual superstructure, ideology plays a very important role in national security, social stability, and healthy economic development. As a result, ideological work is critical to the Party's success, and the current focus of ideological work is to increase ideological risk prevention. The focus of ideological risk avoidance is gradually shifting to cyberspace as the Internet becomes the primary arena and forum for information interchange, value dissemination, and ideological exchanges. Deep learning, as a data processing technology, is characterized by deep data analysis and full generalization and can have an impact on ideological security work: on the one hand, it helps work subjects evaluate and count the process and effect of work in order to grasp the trend of public opinion; on the other hand, it helps work subjects understand and reflect on the inner logic and contemporary value of Marxist theory through diversified work platforms and diverse work methods and promotes work subjects' understanding of Marxist theory. On the other hand, through diversified working platforms and various working methods, we help the working targets to understand and reflect on the inner logic and contemporary values of Marxist theory and promote their true identification with socialist core values. Based on the impact of deep learning on work subjects and work objects, this paper proposes that Marxian ideological security workers can use it to effectively achieve good communication and contemporary value assessment among different work subjects, set specific indicators according to the division of labour, adopt different working methods according to the groups to which the learning bjects belong, and establish a long-term evaluation mechanism in the process.

## 1. Introduction

Along with the accelerated pace of reform and opening, China's economic construction has grown rapidly, and the rapidly changing science and technology has continued to promote economic globalization, and various products from the west have flocked to China [1–3]. In the process of cultural globalization, different national cultures, which are the crystallization of the wisdom of the working people, intermingle and collide with each other. On the one hand, through the continuous exchange and integration of international and local Chinese cultures, we have been able to learn from and appreciate the excellent cultures of different nationalities. On the other hand, the continuous integration of foreign cultures challenges the traditional Chinese culture and has a great impact on the mainstream ideology of China, and various western cultural ideologies impact the ideological consciousness of contemporary college students and affect their ideals and beliefs [2]. Vices such as greed for pleasure and obsession with online games seriously affect the normal study of college students and their desire to pursue ideals and benefit mankind. In today's era, in the face of the great adjustment and change of the world pattern, the frequent intermingling of various ideologies and cultures, and the rise of China, many developed countries are anxious in the international arena, and in the international arena, the western hostile forces are using all available forms to constantly infiltrate and invade China culturally and develop various cultural communication channels to spread their “free thinking” and “hedonism.” They are trying to assimilate China ideologically and culturally by developing various cultural channels of communication and spreading their “free thinking” and “hedonism,” and by propagating their ideology. In China, with the rise of the market economy and the infiltration of western culture, the development of the Chinese cultural market has lagged and is relatively imperfect [4, 5].

RETRACTED

Many young people have become confused about Chinese culture and lack self-confidence in their own outstanding culture, and at the same time, they have become skeptical of the core values of socialism with Chinese characteristics. Some college students are eager to learn about western culture and western festivals and worship everything in the west blindly. Culture carries the future destiny of the nation, and a country and a nation need strong cultural confidence if they want to be invincible in the forest of the world's nations. Cultural confidence is the correct examination and application of the history of the Chinese nation and is the cornerstone of national self-confidence, which must be nurtured in the practice of socialism with Chinese characteristics in the new era. By practicing cultural self-confidence, we can realize the grand blueprint of building a strong cultural nation [6, 7]. The logic of contemporary changes calls for great theories, and great theories keep advancing the emergence of practice. Under the increasingly fierce international competitive environment, studying the cultural self-confidence of college students is an inevitable requirement for realizing a strong cultural nation with Chinese characteristics. Only in this way can the nation have faith, the people have hope, and the country have strength.

RETRACTED

The media industry, communication ecology, and public opinion environment are changing as a result of the iterative development of visual media and the rapid emergence of visual communication, and Internet users' “visual survival” is quietly affecting their cognitive habits and cognitive choices and, even to a degree, their intrinsic value judgment of information [8–10]. The Marxist materialistic dialectic emphasizes that things always have two sides, and it is necessary to grasp them comprehensively from both positive and negative aspects. Therefore, while we are happy to see a wide range of visual landscapes to enrich the online life of Internet users, we must also be aware that many visual information, although superficially no different from other information, contains elements of wrong social trends and antimainstream ideology and implies the realistic purpose of anti-Marxism, and the explosive and fissionable spread of such information is bound to cause ideological erosion to Internet users, leading to a continuous decline in the value of the majority of Internet users. The explosion and fission of this kind of information are destined to produce ideological erosion among netizens, resulting in a steady reduction in the value of most netizens and even a misguided ideological shift. In such circumstances, Internet ideology, as a conceptual superstructure built on an economic foundation, is today facing the hazards of metaphorization [10], fragmentation, and panentertainment, all of which are affecting and contesting mainstream ideology's dominance.  Figure 1 shows the meaning of Marxist philosophy.

Internet users are no longer limited to getting information through old monotonous text media but are increasingly using innovative and dynamic visual media such as photographs and videos, thanks to the iterative updating of mobile information technology. Visual media has arguably become the primary source of information for Internet users [11]. The rise of visual media in cyberspace has not only brought richer and more shocking online life experience for Internet users but also brought new impact and risk to network ideology, which to a certain extent affects the Party's dominance, initiative, and right to speak in network ideology work. The transmutation of the network communication pattern and netizens' access to information requires us to actively explore the use of new technological means to empower ideological work and further enhance the relevance, scientific, and longevity of network ideological risk prevention. As a cutting-edge application of artificial intelligence in the field of vision, visual recognition has the unique ability to intelligently acquire, identify, analyze, and interpret images and video images and is expected to become an important focus point for the innovation of network ideological risk prevention means under the new situation and environment. Therefore, based on the perspective of Marxist theory discipline, this study is dedicated to exploring the important role and realization mechanism of introducing visual recognition in network ideological risk prevention, so as to provide innovative ideas, useful suggestions, and reference paths for the practice of risk prevention in the ideological field as far as possible.

RETRACTED

The organizational paragraph is given below: Section 2 contains the related work.  Section 3 reviews the methods of the proposed work.  Section 4 described the experimental design and results. Finally, the paper ends with the conclusion in Section 5.

## 2. Related Work

### 2.1. Marxist Ideology

Numerous practices have proven that Marxism is a universally applicable reality since the May Fourth Movement and the dissemination of Marx to China. No matter in the war years or in the socialist construction in peacetime [12–14], Marxism has always been a guiding light for the Chinese revolution, and only under the guidance of Marxism can the Chinese revolution be invincible. In the cultivation of cultural self-confidence of college students, adhering to the Marxist view of culture has a double significance. Ideological assessment indicators are shown in Figure 2.

It enriches the theory of cultural self-confidence of college students. Adhering to the Marxist cultural outlook and exploring the cultivation path of cultural confidence of college students not only enrich the connotation of cultural confidence of college students but also expand the theoretical scope of the Marxist cultural outlook. Cultural self-confidence has been mentioned by national leaders many times. Extensive and in-depth discussion on the cultural self-confidence of college students and new initiatives to adapt to the growth of college students under the threshold of Marxist cultural outlook are of great significance to the expansion of the breadth and depth of cultural self-confidence of college students and to the process of advancing Marxist cultural theory, which is not only beneficial to the cultivation of cultural self-confidence of college students but enables also college students to clearly understand the mainstream ideology of Chinese characteristics, which can stimulate the whole nation creativity and innovation of culture [14–16]. Second, it favors the advancement of ideological and political education disciplines in colleges and universities. Adhering to a Marxist view of culture and proposing countermeasures aimed at increasing college students' cultural self-confidence can help to advance and improve college ideological education theory, provide a theoretical foundation for reforming college ideological education, and provide strategies for increasing college students' cultural self-confidence. Adhering to the Marxist cultural view, the discussion on the cultivation of college students' cultural self-confidence is conducive to improving the working methods and approaches of college political education, improving the level of college political education, consolidating the scientific research ability of college political education, and providing strong guarantee for the reform of college political education and the cultivation of talents, which can enhance the timeliness of college students' political education in the new era and strengthen its teaching and education. It can enhance the timeliness of political education for college students in the new era and strengthen the effectiveness of teaching and educating people [17–19]. Third, it demonstrates the profound effect of Marxist cultural perspectives. The discussion on topics connected to the road of nurturing cultural self-confidence among college students can strengthen the theory of Marxist cultural outlook and encourage the greater growth of advanced socialist culture, according to the Marxist cultural outlook. To cultivate the cultural self-confidence of college students, we have a deep cultural heritage and a strong base. The October Socialist Revolution in Russia promoted the progressive intellectuals in China to study and propagate Marxism, and the wide spread of Marxism in China laid the ideological foundation for the establishment of the Communist Party of China, and the Chinese Revolution has had a brand-new guiding ideology and direction since then. Marxist cultural theory is a classic reproduction of human cultural concepts. Starting from a materialistic historical view, it stands at the high point of human culture and reflects the characteristics of the times comprehensively and accurately, “caging heaven and earth within the form and thwarting all things in the brush,” gaining insight into the times, and meeting the light. Nowadays, under the new situation of promoting socialist culture to a higher and deeper goal, adhering to the Marxist view of culture, further analyzing the confusion arising from the cultural self-confidence of college students, finding out where the problems lie, and proposing targeted cultivation programs not only manifest the profound practical logic and theoretical logic of Marxist cultural theory but also make rational thinking and theoretical responses to the cultivation of cultural self-confidence of college students, so that college students can continuously improve their cultural cultivation. It makes college students continuously improve their cultural cultivation [20].

RETRACTED

It is conducive to the transmission of excellent Chinese culture. Guided by the Marxist view of culture, the study of cultural confidence of college students not only helps to inherit and carry forward the excellent Chinese traditional culture but also helps to forge a new splendor of Chinese culture and gives new vitality to the cultivation of enhancing cultural confidence of college students. As the times are changing and the society is changing, college students in the new era should adapt to the development of the times, bear in mind the origin and historical lineage of Chinese national culture, and make efforts to spread it. Only in this way can it be conducive to solving the problems of college students themselves and enhancing the timeliness of Civic Education, and only then can it be conducive to the enhancement of national cultural soft power and influence, strengthening the discourse of the Chinese nation in the international arena, enhancing the international status of the Chinese nation, and showing the style of a great nation for global peace. Second, it is conducive to the formation of a correct life orientation. Educators should appropriately guide college students to determine Marxism's ideology and the wonderful Chinese culture as their knowledge and absorb their comprehensive quality during the university time, which is the formation period of life outlook, world outlook, and values. They should supervise college students to perfect their overall value orientation, improve their cultural literacy, comprehensively strengthen the cultivation of their comprehensive quality, and promote their rational treatment of Chinese and western cultures. We should guide college students to correctly grasp the connotation of mainstream culture, to “look far ahead, be vigilant in peace, be brave in change, be brave in innovation, never be rigid, never be stagnant,” so that under the guidance of Marxist cultural outlook [23], college students can strengthen their cultivation, correct their thinking, not be influenced by western nihilism and retrogressive, and, under the guidance of Marxist cultural outlook, be guided by a loud and clear voice. Under the guidance of the Marxist cultural concept, they will manifest the spiritual power of cultural confidence with a loud main theme and strong positive energy, so that Chinese culture will be more vigorous and vital.

RETRACTED

### 2.2. Deep Learning and Ideology

Metaphor itself is simply a neutral linguistic method that can have both positive and negative effects. However, when metaphors are used in political topics, i.e., when political metaphors are created, they can pose ideological risks and threats. Before the era of visual communication, political metaphors mainly appeared in the form of textual metaphors [16]. However, with the advent of the era of visual communication, a new type of political metaphor, visual metaphor, has emerged quietly, posing a new threat to online ideological security. Visual metaphors refer to the cultural behavior of using visual images such as pictures and videos to suggest people to perceive, imagine, and experience a viewpoint or value. Visual images may seem straightforward and simple, bringing a visual impact without conveying too much of a point of view or value, but they are not. Like words, visual images also can convey ideas and opinions and do so in a more subtle and flexible way. We should not underestimate the power of image cultures, especially dynamic ones, to influence emotions through images and thus to have a significant impact on systems of representation and value. Similarly, visual images are often used as a metaphor, and visual images have an ideology behind them. Therefore, it can be said that the content of visual images is to a large extent ideology and various social trends, which spread and spread in cyberspace by means of visual image shells, so that most Internet users “hear the thunder in silence.” At present, visual metaphors have three main characteristics: first, they spread faster. Visual images have the advantage of being intuitive and dynamic, and their audiences are not restricted by age, region, culture, and occupation, so visual metaphors tend to spread faster and more widely. Second, they are more concealed. In the process of visual metaphors, negative factors are embedded in the visual information structure, which makes them appear calm and untouched on the surface, but in fact, they are treacherous and harmful. Third, it is more attractive. Visual metaphors are often set in the subject matter of interest to Internet users, which can be close to social hotspots and close the distance between the mind and the heart of Internet users, thus attracting them to browse and watch [22-23].

Hostile forces use metaphorical images to attack the mainstream ideology. The characteristics of visual metaphors largely give hostile forces an opportunity to take advantage of them. Hostile Chinese and international forces often target and choose the painful points, hot spots, and focal points of Internet users, especially the youth, and very cleverly express their so-called western “universal values,” neoliberalism and other capitalist ideologies, and wrong social trends with false qualities through visual metaphors. They question the scientific, value, and legitimacy of the mainstream ideology; attack the Party's leadership and the existing institutional arrangement; and vilify the core socialist value system, with the intention of competing with the mainstream ideology for people's hearts and minds. In the communication of visual metaphors, very often, the content expressed by the content distributor does not stop after one simple transmission but is repeatedly transferred and even spread geometrically, so that the undesirable information content is constantly embedded in people's visual neurons, reaches people's minds, and influences their thoughts. Hostile forces are good at infiltrating through uninterrupted and elaborate visual content, like “boiling a frog in warm water” to poison the minds of Internet users, especially the youth, little by little for a long time, in an attempt to achieve the sinister purpose of identifying with their wrong ideas and wrong values. Young Internet users, who are often weak in media literacy, are unwittingly incited and compelled by them, unable to discern between good and evil, resulting in ideological distortion and polarisation. At present, it is very difficult to control such visual metaphors. This is because, for textual metaphors, we can get better control by setting up sensitive words and keywords to retrieve and filter undesirable contents, but not for visual metaphors. The metaphorical connection is not natural but gradually built up during the communication process within the network circle, so it is extremely concealed and creates a more difficult governance problem. This makes it difficult to reach the crux of the problem by using traditional regulation and governance methods, and there is the disadvantage of treating the symptoms but not the root cause, with little effect. At present, almost all mobile social platforms take short videos as the first choice of information dissemination, forming a new pattern of short videos leading and influencing the communication style and content of cyberspace. The biggest feature of short video is to create a “light communication” mode with short duration and small length. This “short” and “light” determine that the content presentation of short videos must be fragmented, fragmentary, and incomplete. Video producers tend to large volume and long content through splicing, editing, compression, and other techniques to process and then produce a short video; a few minutes of content is often cut from several minutes or even hours of content. This content fragmentation problem is characterized by the commonality of short videos and the performance of many objects, and the effect is not the same. For the expression of life and leisure content, short video is the most suitable media tool. This is because the content of life and leisure does not seek to express the complete, logical, rational thinking, but the most important thing is to express the emotion; the most important thing is to be concise; the most important thing is to go straight to the subject; short video is suitable for this demand. For example, using short videos to watch TV series, movies, and variety shows can help Internet users with limited free time to focus on the main plot of the TV series, movies, and variety shows; using short videos to watch sports highlights can help Internet users who miss the opportunity to experience live games to quickly view the highlights afterwards. However, for serious content and theoretical content, short videos add to the difficulty of expression, making it difficult to present the original content in a panoramic view and accurately express the true and perfect meaning of mainstream ideology.

RETRACTED

## 3. Methods

In this section, we defined the model structure, data preprocessing, text features, word embedding, LSTM layer, and output layer in detail.

### 3.1. Model Structure

Traditional machine learning, according to previous research, always suffers from the problem that the influence of Marxian ideology recognition is restricted by the corpus size and feature selection, resulting in a lack of generalization ability in complicated recognition tasks. To address the above problems, a hybrid deep neural network-based sentiment recognition model for Chinese Marxian ideology text is proposed through the study of deep learning, as shown in Figures 3. The model integrates bi-LSTM, CNN, and with attention mechanism, which first obtains the contextual semantic features of the corpus and then extracts local semantic features, while giving r different schemes of attention to the feature information at each moment in order to get a better representation of text features and then further improve the accuracy of text sentiment recognition.

The model mainly consists of seven parts:

1. Input layer: acquisition of corpus data
2. Preprocessing layer: splitting words and removing irrelevant data
3. Bi-LSTM layer: extracting contextual semantic features of the corpus
4. Attention mechanism layer: obtaining weighted contextual semantic features with different focus representations of the sentence
5. kCNN layer: obtaining the final vector representation containing both contextual and local semantic features
6. Output layer: realize text recognition prediction

The steps are briefly described as follows:

1. Obtain real text corpus data through crawlers and other means
2. Preprocessing of the corpus such as word separation
3. Vectorized representation of the corpus text:
4. Build a Chinese text sentiment recognition model based on hybrid deep neural network
5. Designing the cost function and training the network with relevant algorithms
6. Validation of the model using the validation set corpus
7. Practical application of the model

RETRACTED

### 3.2. Data Preprocessing

#### 3.2.1. Text Corpus Cleaning Preprocessing

The main purpose is to carry out traditional and simplified conversion and remove duplicate data and irrelevant data in the Marxian ideological corpus, involving special symbols, text, HTML web tags, and other processing objects. The duplicate data may be the result of wrong crawling in the process of crawling data or due to the malicious brush reviews of the network water army; whatever the reason is, the same data need to be filtered. The original corpus sometimes also contains some meaningless text data, such as text content is full of numbers, letters, symbols, etc. This kind of corpus usually does not have much emotional information. If we do not filter out the repetitious and irrelevant data, it will inevitably impair the recognition effect, and these two types of data can be processed using Excel and other ways. The corpus is labeled with categories, such as good, medium, and bad reviews. The corpus is divided into words and deactivated using jieba. It is the process of cutting the text in the corpus into a series of sentences based on punctuation and then cutting the sentences into individual words, and it is found that the effect of precise mode of word separation is relatively good. Since some new Internet terms usually appear in the web text and the content is often colloquial, it is often necessary to load the user dictionary in order to make the word separation more accurate. User dictionaries are composed of unregistered words, user-built dictionaries, etc. In the user-built dictionaries, some domain-specific terms can be organized. The identification of unregistered words can be achieved by using fastText new word discovery algorithm, adding them to the user dictionary, then using sentiment polarity calculation algorithm to determine their sentiment polarity, and then adding them to the semantic sentiment dictionary if they are sentiment words. In addition, some common deactivated words should be removed in this process; most of them are some auxiliary words, tone words, and some symbols, which not only do not provide help but also take up resources making the processing time grow. The removal of deactivated words can be done through the constructed deactivated word lexicon. To make the model work well for long text data, the corpus is further filtered with the TextRank algorithm to avoid the problem of “dimensional disaster” in the subsequent processing, the preprocessed corpus is divided into three parts: validation set, test set, and training set.

RETRACTED

### 3.3. Text Features

In this paper, a new algorithm TextRank is used to achieve text feature extraction. The algorithm comes from the PageRank algorithm, which is a graph-based algorithm for calculating the importance ranking of web pages; it treats the whole network as a graph; the nodes are web pages; if there is a link relationship between two nodes, then there will be an edge between these two nodes. The importance of the pages *S*(*V*) is

(1) $$\begin{array}{c} S\left(V_{i}\right)=\left(1-d\right)+d*\underset{j\in \ln\left(v_{i}\right)}{\sum }\;\frac{S\left(V_{j}\right)}{\left|\text{Out}\left(V_{j}\right)\right|}, \end{array}$$

where *d* is the damping factor used for smoothing, *S*(*V*_*j*_) indicates the existence of a collection of web pages pointing to the web page; links, Out(*V*_*j*_) indicates the collection of web pages to which the web page *V*_*j*_ can jump, and |Out(*V*_*j*_)| is the number of elements in the collection. The inspiration from the study of the PageRank algorithm is that for text, as long as the graph can be constructed from words/sentences, and then, the relationships between nodes in this graph can be determined by some method, such as word order relationships, semantic relationships, and content similarity; then, we can use the PageRank algorithm to get the core information such as keywords and key sentences in the corpus. Using sentences as nodes, we construct edges with the similarity relationship *S*(*S*_*i*_, *S*_*j*_) between sentences.

(2) $$\begin{array}{c} S\left(S_{i},S_{j}\right)=\frac{\left|\left\{w_{k}\left|w_{k}\in S_{i}\&w_{k}\in S_{j}\right.\right\}\right|}{\log\left(\left|S_{i}\right|\right)+\log\left(S_{j}\right)}. \end{array}$$

Iterate the node weights until convergence; sort the node set weights in reverse order, and output the most important *N* results.

### 3.4. Word Embedding

In order to enable the computer to recognize and process Marxian ideological text content, the corpus first needs to be converted into digital form. The text data *T* with labels are loaded by batch, and then, the word embedding matrix E obtained by Word2Vec is mapped to map the text *T* containing the comment content *D* and the label content *L* into a three-dimensional vector matrix E. At this point, a vectorized text *T*_*j*_ = {*x*_1_, *x*_2_, ⋯, *x*_*i*_, ⋯, *x*_*n*_} containing n words denote *E* is described as follows:

(3) $$\begin{array}{c} E=\left(e_{1},e_{2},\cdots ,e_{i},\cdots ,e_{n}\right),\\ e_{i}=w_{x_{i}}E_{\text{w}}, \end{array}$$

where *E* ∈ *R*^batch×Sxdd^, *E*_*V*_ ∈ *R*^*V*_*n*_×*d*^, batch is the size of the batch data, *S* is the set text sequence threshold, *d* is the word vector dimension, *V*_w_ denotes the word embedding matrix size, and *w* is the index of the one-to-one correspondence between word *x* and *E*. The flow chart of text vectorization is shown in Figure 4.

RETRACTED

### 3.5. LSTM Layer

When LSTM extracts the contextual semantic features of the text, the cell information at moment t is updated as follows:

(4) $$\begin{array}{c} i_{\text{t}}=\sigma \left(W_{\text{ei}}e_{\text{t}}+W_{\text{hi}}h_{\text{t}-1}+b_{\text{i}}\right),\\ f_{\text{t}}=\sigma \left(W_{\text{ef}}e_{\text{t}}+W_{\text{hf}}h_{\text{t}-1}+b_{f}\right),\\ g_{\text{t}}=\tanh\left(W_{\text{ec}}e_{\text{t}}+W_{\text{hf}}h_{\text{t}-1}+b_{\text{c}},\right),\\ c_{\text{t}}=i_{\text{t}}g_{\text{t}}+f_{\text{t}}c_{\text{t}-1},\\ o_{\text{t}}=\sigma \left(W_{\text{eo}}e_{\text{t}}+W_{\text{ho}}h_{\text{t}-1}+b_{\text{o}}\right),\\ h_{\text{t}}=o_{\text{t}}\tanh\left(c_{\text{t}}\right), \end{array}$$

where *i*_t_, *f*_t_, *o*_t_, and *g*_t_ denote input gate, forget gate, output gate, and candidate gate, respectively; *W*_ei_, *W*_hi_, *W*_ef_, *W*_hf_, *W*_ec_, *W*_eo_, *W*_ho_, and *W*_hf_ denote weights; and *σ* and tanh are activation functions. However, LSTM only focuses on the temporal information and ignores the most important contextual information in the text. Bi-LSTM extends the one-way LSTM into a bidirectional structure, which retains the good performance of LSTM and can obtain the pre- and postcontextual information well. Input *E* into the forward and backward structures of bi-LSTM, respectively, to get the forward and reverse hidden features, and the cascade is the output *h* at the *i*th moment, and finally, the output of each moment is spliced to get the contextual semantic features.

(5) $$\begin{array}{c} H=\left(h_{1},h_{2},\cdots ,h_{\text{i}}\cdots ,h_{\text{n}}\right),\\ h_{\text{i}}=\left[{\overset{⟶}{h}}_{\text{i}}⊕{\bar{h}}_{i}\right], \end{array}$$

where *H* ∈ *R*^batch×*n*×2*d*^, ⊕ is the splicing process, and *n* is the required time size and equal to the text sequence threshold.

### 3.6. Output Layer

Inputting *C* to the output layer, the output vector *p*(*y*) is obtained by determining the class to which the Marxian ideological text belongs through SoftMax. To prevent overfitting, the dropout technique, a common measure in neural network models, is used in this layer.

(6) $$\begin{array}{c} p\left(y\right)=\text{soft}\max\left(W_{c}C_{d}+b_{c}\right), \end{array}$$

where *p*(*y*) ∈ *R*^hatchixclasses^; *W*_*c*_ ∈ *R*^2*n*×*c* lasses^ and *b*_*c*_ are the weight matrix and bias matrix of the output layer, respectively; and classes are the number of recognition categories required by the task. Softmax is used to estimate the probability *p*(*v*) that the corpus text belongs to each target recognition category, and the label corresponding to the maximum probability *y* is selected from it as the final recognition. The result is selected as the final recognition result.

(7) $$\begin{array}{c} y=\arg\max\left(p\left(y\right)\right). \end{array}$$

In this paper, when training the model, the cost function *J*(*θ*) is used as the crossentropy between the output of the model and the corpus labels, and the model parameter *e* is updated using the Adam optimizer with good performance in deep learning, and the training process is shown in Figure 5.

(8) $$\begin{array}{c} J\left(\theta \right)=\frac{1}{N}E\left(D,L;\theta \right)+\frac{\lambda }{2}{\left\|\theta \right\|}^{2},\\ E\left(D,L;\theta \right)=-\overset{N}{\underset{i=0}{\sum }}\;\left\{p\left(L_{\text{i}}\right)\log\left(y;\theta \right)+\left[1-p\left(L_{\text{i}}\right)\right]\log\left[1-\left(y;\theta \right)\right]\right\}. \end{array}$$

RETRACTED

## 4. Experiments and Results

In order to ensure the objectivity and authenticity of the experiment, the corpus used in this experiment was crawled using crawler technology to crawl the comment data about Marx's ideology-related content on a large Chinese social platform, and the basic information of the corpus is shown in Table 1, and Figure 6 shows the sentence length distribution of the corpus.

The experiment is implemented in TensorFlow deep learning framework using Python language and the specific experimental environment configuration.  Table 2 shows that the experimental findings indicate good performance in both general and particular recognition outcomes for each category. The model also has higher recognition accuracy in real estate, lottery, finance, sports, and gaming, but lower recognition accuracy in society, science and technology, and other fields. The latter may be related to the constant emergence of new words and the rapid changes of current affairs and social hotspots, while new topics and new terms may not be recognized in time for the model that has been trained, so the performance in these fields will be slightly worse.

RETRACTED

The results of the ablation experiments are shown in Table 3. As can be seen from Experiments 20 and 21, the *F*-value of bi-LSTM is improved by about 3% compared with LSTM, which indicates that bi-LSTM with two-layer network structure of forward and reverse can better obtain the contextual information of the text, so the accuracy will be improved, but the complexity is greater than that of LSTM network, resulting in a slightly longer computing time compared with LSTM. As can be seen from Experiments 21 and 22, using the attention mechanism after the bi-LSTM model leads to an improvement in the *F*-value of about 4%, which indicates that attention does have the ability to identify key information that can be helpful for the results. Due to the unique model parameter-sharing feature of CNN, it makes the recognition effect not the best, but it can greatly save the computing time. Experiments 19-23 show that the RCNN network, which combines the advantages of RNN (and its variants) and CNN, outperforms each network individually. From the whole Table 3, the network model proposed in this section has the highest accuracy, which indicates that the deep neural network obtained by integrating bi-LSTM and CNN and introducing the attention mechanism, using TextRank algorithm in the preprocessing process, and using dropout technique in order to avoid overfitting, L2 regularization, and early stopping three strategies is a very effective method for Chinese text sentiment recognition.

## 5. Conclusion

Marxism believes that society is constantly changing, developing, and moving forward. Ideological work must always adhere to the materialistic view of history, problem-oriented, advancing with the times, deepening understanding with the development of the times, constantly innovating ideas, and constantly updating the means. In this sense, the network ideological risk prevention is only a work in progress; there is no time to complete; we cannot let down our guard; we must rely closely on new technological means to manage the network, especially the application of artificial intelligence to help network ideological work, to ensure that cyberspace adhere to the correct, mainstream orientation of public opinion and value orientation. Looking ahead, the new wave of technology, which has artificial intelligence at its core, will continue to make significant progress. Visual recognition technology will also usher in new iterations of upgrading opportunities, and we have reason to believe that the strong leadership of the Party, as well as the joint participation of multiple subjects, will help to accelerate this process. Artificial intelligence-supported network is a good technique to ensure that the network ideological risk prevention work to introduce the role of visual recognition will continue to improve. Work on preventing ideological risk will be more steady and widespread, and the Internet will be brighter, cleaner, and clearer.

RETRACTED

## Figures and Tables

**Figure 1:** Marxist theory connotation.

**Figure 2:** Ideological assessment indicators.

**Figure 3:** Model architecture.

**Figure 4:** Text vectorization.

**Figure 5:** Training process.

**Figure 6:** Sentence length distribution of the corpus.

**Table 1:** Corpus information.

Category	Good reviews (5 stars)/article	Moderate rating (3 stars)/article	Poor reviews (1 star)/article
Training set	600	600	600
Test set	150	150	150
Validation set	100	100	100

**Table 2:** Performance comparison.

Models	Number of cycles	Training time (s)	Test time (s)	Accuracy rate	Recall rate	F1 value
CNN	3800	3594	36	0.89	0.89	0.89
LSTM	2300	33456	139	0.77	0.77	0.76
Bi-LSTM	4000	219008	1412	0.88	0.87	0.87
Bi-LSTM-attention	4000	206272	776	0.90	0.90	0.90
RCNN	1900	185709	2051	0.92	0.91	0.91
Proposed method	5000	162950	720	0.94	0.94	0.94

**Table 3:** Results of ablation experiments.

Models	*P*	*R*	F1
SVM + Word2vec + wordiness + adverb of degree + emotion + negation	0.88	0.78	0.81
SVM + Word2vec + transitive + wordiness + degree adverb + emotional word + negative word	0.89	0.86	0.88
SVM + Word2vec + conditionals + transitions + wordiness + degree adverbs + emotional words + negation	0.90	0.91	0.90
SVM + Word2vec + punctuation + conditional word + transitive + degree adverb + negative word + emotional word + negative word	0.86	0.88	0.85
NB + Word2vec + word vector averaging	0.76	0.74	0.75
NB + Word2vec + word vector^“^voting^”^ method	0.77	0.82	0.80
NB + Word2vec + emotional words	0.98	0.96	0.99

## Data Availability

The datasets used during the current study are available from the corresponding author on reasonable request.
